# Analysis of Structured Data in Biomedicine Using Soft Computing Techniques and Computational Analysis

This article has been retracted.

**DOI:** 10.1155/2022/4711244

**Published:** 2022-10-10

**Authors:** Yanping Wu, Md. Habibur Rahman

**Affiliations:** ^1^Hangzhou Medical College, Hangzhou 311399, China; ^2^Department of Information and Communication Technology, Bangabandhu Sheikh Mujibur Rahman Digital University Bangladesh, Gazipur 1750, Bangladesh

## Abstract

In the field of biomedicine, enormous data are generated in a structured and unstructured form every day. Soft computing techniques play a major role in the interpretation and classification of the data to make appropriate decisions for making policies. The field of medical science and biomedicine needs efficient soft computing-based methods which can process all kind of data such as structured data, categorical data, and unstructured data to generate meaningful outcome for decision-making. The soft-computing methods allow clustering of similar data, classification of data, predictions from big-data analysis, and decision-making on the basis of analysis of data. A novel method is proposed in the paper using soft-computing methods where clustering mechanisms and classification mechanisms are used to process the biomedicine data for productive outcomes. Fuzzy logic and C-means clustering are devised as a collaborative approach to analyze the biomedicine data by reducing the time and space complexity of the clustering solutions. This research work is considering categorical data, numeric data, and structured data for the interpretation of data to make further decisions. Timely decisions are very important especially in the field of biomedicine because human health and human lives are involved in this field and delays in decision-making may cause threats to human lives. The COVID-19 situation was a recent example where timely diagnosis and interpretations played significant roles in saving the lives of people. Therefore, this research work has attempted to use soft computing techniques for the successful clustering of similar medical data and for quicker interpretation of data to support the decision-making processes related to medical fields.

## 1. Introduction

### 1.1. Background

Data mining is to process where hidden information is retrieved from complex data sets by interpreting the data in an appropriate way [1]. With the increasing use of digital technology in biomedical applications, such as electronic biomedical records and digital imaging technologies, large volumes of biomedical data are collected daily [2]. The plenty of stored biomedical data has led to an urgent request for new methods and tools to transform the accumulated data into readable biomedical information [3]. This has opened up exciting opportunities for the application of data mining techniques to develop new prediction and diagnosis models in biomedicine. Clustering is an important technique in data mining to partition a set of data objects into subsets according to data similarity [4]. Similar data are placed in one cluster. The clustering technique has been applied widely in biomedicine [5]. There are several complexities of biomedical data that challenge the application of clustering techniques in biomedicine. The first challenge is the ambiguity of biomedical data caused by the fact that one feature might be an indicator for two or more clusters with similar attributes or that certain features are not explicitly recorded in biomedical records [6]. This ambiguity can cause an overlap of cluster boundaries, i.e., the same class of feature may belong to several biomedicine clusters. In the traditional clustering technique, a hard-clustering method is used to arbitrarily partition a class of features into one cluster. Although this hard clustering method eliminates ambiguity, it can also cause information loss of that feature as an indicator for another cluster [7]. Therefore, the traditional clustering technique is suboptimal and there is a need for newer techniques. The fuzzy clustering algorithm (FCM), a specific type of clustering technique, has been introduced to resolve this challenge, arising from the ambiguity of biomedical datum, by partitioning data according to fuzzy membership values. Fuzzy membership is the data's degree of similarity with each cluster. As one piece of data may have varying degrees of similarity with several clusters, a fuzzy clustering algorithm uses iterative algorithms, such as objective function, to compute the membership of the data into several relevant clusters with varying membership values. The FCM clustering algorithm is a specific type of fuzzy clustering algorithm developed by Bezdek [5]. For objective function, the FCM algorithm assigns a fuzzy membership value between 0 and 1 to each data object according to the data's distance to a cluster center. The notion of “fuzzy” implies that a data's membership is not fixed, but dynamic in association with its varying distance to different clusters. For example, as the symptom of chest pain can be an indicator for both congestive heart failure and chest injury, its membership to the congestive heart failure cluster can be 0.5, and to the heart failure cluster can be 0.3. Only after the possibility of chest injury is completely eliminated according to X-ray scanning results can the membership of this symptom be entirely associated with congestive heart failure. Due to its ability to handle the “fuzzy” nature of biomedical data, the FCM algorithm has been widely applied in biomedicine for such things as disease detection, biomedical image segmentation, and biomedical feature selection [8]. To date, the biggest challenge for the FCM algorithm remains how to handle the complexity of biomedical data including both categorical data (e.g., name, group) and numeric data (e.g., time, length) [9]. This shows a more realistic and accurate approach for clustering the medical data.

### 1.2. Literature Review

In reference [10], the authors state that different representations, processing, and computation are required for numeric and categorical data. The traditional method of using an objective function to directly measure the Euclidean distance for clustering numeric data would not work for categorical data, which does not have explicit Euclidean distance. To deal with this challenge, two methods have been widely used to convert different types of biomedical data. One is to convert the categorical data into numerical data using a binary coding technique, i.e., coding “yes” as “1,” and “no” as “0.” Another method is to convert numeric data into categorical data by a discretization method. For example, this might convert length into three groups, those aged between “20 to 30” as “1,” “30 to 40” as “2,” “40 to 50” as “3,” and so on. It is no surprise that with a process as complicated as data conversion, problems emerge throughout the process. One of the common problems with data conversion is losing information. For example, if converting length “20 to 30” to “1,” the useful information may be lost that the characteristics for the length group of 20 to 25 are significantly different from that of the 25 to 30 group. In reference [11], the researchers propose an algorithm to directly cluster categorical biomedical data. For example, Huang et al. designed a k-prototypes algorithm by combining k-means and k-modes algorithms to directly cluster categorical data without conversion. In reference [12], the authors assess different clustering techniques. Data clustering techniques can be of two types: partitioning procedures and hierarchical procedures. The first one creates a hierarchy of clusters. The results are shown as a dendrogram. Partitioning method-clustering makes various partitions of objects and evaluates them by some standard. In reference [13], the authors provide biomedical researchers with an overview of the status quo of clustering algorithms. They also illustrate examples of biomedical applications based on cluster analysis. The research helps to select the most suitable clustering algorithm for different types of applications. In reference [14], the authors propose a novel method for clustering and analysis of complete biomedical article texts. The cosine coefficient is used on a subspace of two vectors. The Euclidean distance is not computed for all vectors. Then, a strategy and algorithm are introduced for semi-supervised affinity propagation (SSAP). The results show that the SSAP outperforms conventional k-means methods. In reference [15], A similarity-based agglomerative clustering (SBAC) algorithm is used to cluster data by similarity to reach a cohesive hierarchical cluster. In reference [16], a modified FCM clustering technique with a hybrid fuzzy time series model is used to deal with disease interval information to predict the infected cases and deaths of COVID-19. Some authors put forward the Kullback–Leibler FCM algorithm to process Gauss-multinomial-distributed data sets (KL-FCM-GM) [17]. In reference [18], the authors have applied a firefly algorithm in the objective function for cluster center selection. By combining the first step of cluster center selection with the second step of calculating the objective function, this algorithm effectively overcomes the limitation of local cluster optimization, and thus was useful for clustering a large medical data set [19].

### 1.3. Contribution of the Paper

- The Fuzzy C-means (FCM) clustering algorithm has been proposed to analyze biomedical datasets in this paper by adding a weighted mechanism. This study proposes a novel multiple weighted Fuzzy C-means for Mixed Data (MD-MWFCM) clustering algorithm.
- The MD-MWFCM algorithm presents a novel clustering FCM algorithm by treating numeric and categorical data individually with their respective cluster center representation, dissimilarity measurement, and objective function aspects.
- The model is proposed that will take care of numerical and categorical data.
- The performance of the MD-WFCM algorithm has illustrated its useful application not only in a pure attribute dataset (numerical data or categorical data) but also, more importantly, in a mixed biomedical dataset.
- The MD-MWFCM algorithm is improved from cluster center initialization through the minimum threshold method.

## 2. Proposed Methodology

### 2.1. FCM Algorithm

There are three common data processing steps in applying the FCM algorithm:

  Step 1: initializing the cluster centers and fuzzy membership matrix.
  Step 2: calculating the objective function and update the cluster centers.
  Step 3: continuously iterating through Steps 1 and 2 until the defined threshold of the membership cluster is reached.

One of the limitations of the FCM algorithm was, that it is oversensitive to the location of cluster centers initialized in Step 1. The selection of a cluster center is vital because the center is used by the objective function to calculate the Euclidian distance of a data point. Previous researchers have developed various methods to optimize the selection of cluster centers. Another limitation of the FCM algorithm is no discretion of the varying weights of an attribute in different clusters in Step 2. This may cause limitations for the FCM to reach an appropriate level of performance in clustering biomedical data. A data attribute was assumed to have the same weight in different clusters, which is not always the case for biomedical data. This leads to the same dissimilarity measurement used to process both numeric data and categorical data without considering the differences between the two data sets, which may cause the loss of biomedical information. The optimal algorithm would be to analyze the data in its original data format.

To improve this method, some researchers such as Xiao et al. have tried proposing a Gaussian smoothed and weighted FCM clustering algorithm (WGFCM) in brain magnetic resonance image segmentation [19]. Improvements have been made on certain aspects of FCM, i.e., optimization of initial cluster centers and assignment of weights of an attribute to various cluster centers [20]. Smart technologies have also implemented several information extraction methods in artificial intelligence, internet of things, cyber-physical system, cybersecurity and so on [21]. One of the data mining algorithms quantum adaption cuckoo search (QACS) is used to identify the unauthorised users by extracting the important features in blockchain technology [22]. However, there is a need for an effective method and process in clustering mixed numerical and categorical data for the biomedical data set. To address this challenge, we propose a novel multiple weighted Fuzzy C-means for mixed data (MD-MWFCM). Instead of data transformation, the MD-MWFCM will improve data representation by directly using the original data type for clustering analysis. It will use different dissimilarity measurement methods to treat different data types and then calculate the distance of a data point with weighting to various cluster centers. Different methods will be used to represent cluster centers for different data types; mean will be used for numeric data and fuzzy center will be used for categorical data. This will lead to improvement in the selection of the initial cluster center.

### 2.2. The MD-MWFCM Algorithm

k-Means is a widely used algorithm for clustering. Its limitation is that it only works for numerical data. It is not suitable for categorical data types. Modified variation is k-Modes which is created in order to handle clustering algorithms with the categorical data type. The limitation of k-mode is that it can handle categorical data only. The proposed algorithm can handle numerical as well as categorical data. Mean will be used for numeric data and fuzzy center will be used for categorical data. This will lead to improvement in the selection of the initial cluster center.

The proposed method also introduces a cluster initialization strategy in which the attributes have been assigned weights. The attribute domains include both numeric and categorical domains. A new method is proposed to measure the similarity level between the value of a categorical attribute of the variable to the center of a categorical cluster . It is based on a method proposed in the article [7]. Binary distance *δ*(*x*_*ij*,*a*_*kj*^*t*) is used to measure the similarity between the variable and cluster center. The resulting value of *δ*(*x*_*ij,a_kj*^*t*) is between 0 and 1 depending on the level of similarity between the variable and cluster center. This will lead to improvement in the selection of the initial cluster center.

#### 2.2.1. Data Notation

Let *X*={*X*_1_, *X*_2_, ⋯, *X*_*n*_} denote a set of *n* data points to be clustered and *X*_*i*_(*i*=1, 2, ⋯, *n*) be a data point with *m* attributes {*A*_1_, *A*_2_, ⋯, *A*_*m*_}. Each attribute *A*_*j*_(*j*=1, 2, ⋯, *m*) includes a domain of values denoted by Dom(*A*_*j*_). A data point *X*_*i*_ can be expressed with attributes as in equation (1) as follows:

(1) $$\begin{array}{c} \left[A_{1}=x_{i1}\right]⋀\left[A_{2}=x_{i2}\right]⋀\cdots ⋀\left[A_{j}=x_{ij}\right]\cdots ⋀\left[A_{m}=x_{im}\right], \end{array}$$

where *x*_*ij*_ ∈ Dom(*A*_*j*_) for *j*=1, 2, ⋯, *m*. Values to the set of attribute weights are given in equation (2) as follows:

(2) $$\begin{array}{c} W={\left[w_{1},w_{2},\cdots ,{w_{j},\cdots ,w}_{m}\right]}^{T}\text{,}\\ \forall j:w_{j}>0,\overset{m}{\underset{j=1}{\sum }}w_{j}=1\text{.} \end{array}$$

The attribute domains include both numeric and categorical domains. The categorical domain is denoted by Dom(*A*_*j*_)={*a*_*j*_^1^, *a*_*j*_^2^, ⋯, *a*_*j*_^*n*_*l*_^}, where *n*_*l*_ is the value number of a categorical attribute *j*. *X*_*i*_ is represented as a vector. It represents the data points to be clustered. The same is given in equation (3) as follows:

(3) $$\begin{array}{c} X_{i}=\left[x_{i1}^{r},x_{i2}^{r},\cdots ,x_{ip}^{r},x_{i\left(p+1\right)}^{c},x_{i\left(p+2\right)}^{c},\cdots ,x_{im}^{c}\right]\left(i=1,2,\cdots ,n\right)\text{,} \end{array}$$

where elements *p* with superscript *r* and *p* with superscript *c* are numeric values and categorical values, respectively, and each *X*_*i*_(*i*=1, 2, ⋯, *n*) with *m* attributes. The attribute weight is represented in equation (4).

(4) $$\begin{array}{c} W={\left[w_{1}^{r},w_{2}^{r},\cdots ,w_{p}^{r},w_{\left(p+1\right)}^{c},w_{\left(p+2\right)}^{c},\cdots ,w_{m}^{c}\right]}^{T}\text{.} \end{array}$$

#### 2.2.2. Fuzzy Centre for Categorical Data

A set of n data points *X*={*X*_1_, *X*_2_, ⋯, *X*_*n*_} have both numeric and categorical attributes. They belong to *C* clusters. Their corresponding cluster center set is calculated in equation (5) as follows:

(5) $$\begin{array}{c} V=\left[V_{1},\cdots {,V}_{k},\cdots ,V_{c}\right]\left(k=1,2,\cdots ,C\right)\text{.} \end{array}$$

Each cluster center *V*_*k*_(*k*=1, 2, ⋯, *C*), includes numeric and categorical attributes and can be represented equation (6) as follows:

(6) $$\begin{array}{c} V_{k}=\left[v_{i1}^{r},v_{i2}^{r},\cdots ,v_{ip}^{r},v_{i\left(p+1\right)}^{c},v_{i\left(p+2\right)}^{c},\cdots ,v_{im}^{c}\right]\text{,} \end{array}$$

where elements *p* are defined in equation (3). Every cluster center *V*_*k*_(*k*=1, 2, ⋯, *C*) has exactly *m* attributes. For each of the categorical data of the mixed data set *X*_*k*_^*c*^=[*X*_*i*(*p*+1)_^*c*^, *X*_*i*(*p*+2)_^*c*^, ⋯, *X*_*im*_^*c*^], there exist *C* fuzzy centers $V_{k}^{c}{=\tilde{v}}_{k}\left(k=1,2,\cdots ,C\right)$ [5]. For a fuzzy center ${\tilde{v}}_{k}\left(k=1,2,\cdots ,C\right)$ in the categorical data domain Dom(*A*_*j*_)={*a*_*j*_^1^, *a*_*j*_^2^, ⋯, *a*_*j*_^*t*^, ⋯, *a*_*j*_^*n*_*l*_^}, the fuzzy center of the categorical data set, denoted by $\tilde{V}$, is defined in equations (7) as follows:

(7) $$\begin{array}{c} \tilde{V}=\left[{\tilde{v}}_{1},\cdots {\tilde{v}}_{k},\cdots ,{\tilde{v}}_{c}\right]\left(k=1,2,\cdots ,C\right)\text{,}\\ {\tilde{v}}_{k}=\left[{v_{i\left(p+1\right)}^{c},v}_{\left(ip+2\right)}^{c},\cdots ,v_{im}^{c}\right]\text{.} \end{array}$$

The cluster center ${\tilde{v}}_{k}^{c}$ of the categorical attribute *j*(*j*=(*p*+1), (*p*+2), ⋯, *m*) is as in equation (8):

(8) $$\begin{array}{c} v_{kj}^{c}=\frac{a_{j}^{1}}{\omega_{kj}^{1}}=+\frac{a_{j}^{2}}{\omega_{kj}^{2}}+\cdots +\frac{a_{j}^{t}}{\omega_{kj}^{t}}+\cdots +\frac{a_{j}^{n_{l}}}{\omega_{kj}^{n_{l}}}\text{,} \end{array}$$

where *ω*_*kj*_^*t*^ is subject to the condition given in equation (9).

(9) $$\begin{array}{c} 0\leq \omega_{kj}^{t}\leq 1,\overset{n_{l}}{\underset{t=1}{\sum }}\omega_{kj}^{t}=1,\left(j=\left(p+1\right),\left(p+2\right),\cdots ,m\right)\text{.} \end{array}$$

The cluster center ${\tilde{v}}_{k}^{c}$ of the categorical attribute *j* can be deduced in equation (11) as follows

(10) $$\begin{array}{c} v_{kj}^{c}=\overset{n_{l}}{\underset{t=1}{\sum }}\frac{\sum_{i=1}^{n}1\left(x_{ij}=a_{j}^{t}\right){\left(\mu_{ik}\right)}^{\alpha }}{\sum_{i=1}^{n}{\left(\mu_{ik}\right)}^{\alpha }}a_{j}^{t}\left(j=\left(p+1\right),\left(p+2\right),\cdots ,m\right)\text{,} \end{array}$$

where *n*_*l*_ is the value number of a categorical attribute *j*, *t* is the *t*(*t*=1, 2, ⋯, *n*_*l*_) value of a categorical attribute *j*, *μ*_*ik*_ indicates the fuzzy membership degree of data *X*_*i*_(*i*=1, 2, ⋯, *n*) to the *k* th(*k*=1, 2, ⋯, *C*)cluster. *μ*_*ik*_ is an element of the partition matrix *U*_*n*×*c*_, and subject to condition given in equation (11) as follows-

(11) $$\begin{array}{c} \overset{C}{\underset{k=1}{\sum }}\mu_{ik}=1,0\leq \mu_{ik}\leq 1\text{.} \end{array}$$

Each attribute has a fuzzy categorical value ${\tilde{v}}_{j}\in \tilde{V}\text{ ,}$ represented as a fuzzy set {(*a*_*j*_^*t*^, *ω*_*j*_^*t*^)}(*t*=1, 2, ⋯, *n*_*l*_). The parameter *α*, the fuzzy coefficient exponent, controls the fuzzy degree of partition matrix *U* ∈ *R*^*C*×*n*^. According to previous experience, for numbers in clusters 2–10, the best choice for *α* is from 1.01 to 7.0.

#### 2.2.3. Similarity Level between Two Categorical Attributes

Let *x* denote categorical data and *y* be the cluster center of *x*. The previous studies measure the similarity between *x* and *y* with function *δ*(*x*, *y*). This has resulted in the “hard partition” of *x* into only one categorical cluster *y* if *x*=*y* or vice versa if *x* ≠ *y*. Namely, $\delta \left(x,y\right)=\left\{\begin{array}{c} 0,x\neq y\\ 1,x=y \end{array}\right.\text{.}$ A new method is proposed to measure similarity level between the value of a categorical attribute *x*_*ij*_ of the *j*^*th*^ variable to the center of a categorical cluster *a*_*kj*_^*t*^ based on a method proposed in article [7]. We use binary distance *δ*(*x*_*ij*_, *a*_*kj*_^*t*^) to measure similarity between *x*_*ij*_ and *a*_*kj*_^*t*^(1 ≤ *t* ≤ *n*_*l*_). The resulting value of *δ*(*x*_*ij*_, *a*_*kj*_^*t*^) is between 0 and 1 depending on the level of similarity between *x*_*ij*_ and *a*_*kj*_^*t*^. The similarity function is stated as follows in equation (12).

(12) $$\begin{array}{c} \delta \left(x_{ij},a_{kj}^{t}\right)=\frac{1}{C}\left(\overset{C}{\underset{k=1}{\sum }}\left|\frac{N_{x_{ij},k}}{N_{x_{ij}}}-\frac{N_{a_{kj}^{t}}}{N_{a_{j}^{t}}}\right|\right), \end{array}$$

where *N*_*x*_*ij*_,*k*_ is the data number in dataset *X*_*i*_(*i*=1, 2, ⋯, *n*) with the value *x*_*ij*_ for the *j*^*th*^(*j*=(*p*+1), (*p*+2), ⋯, *m*) attribute of the cluster *k*(*k*=1, 2, ⋯, *C*). With the fuzzy membership (*μ*_*ik*_)^*α*^ of the data point *x*_*ij*_, we can compute *N*_*x*_*ij*_,*k*_, the association of value *x*_*ij*_ for *j*^*th*^ attribute within cluster *k*. The data number in dataset *X*_*i*_ is calculated in equation (13) as follows:

(13) $$\begin{array}{c} N_{x_{ij},k}=\overset{n}{\underset{l=1,l\neq i}{\sum }}1\left(x_{lj}=x_{ij}\right){\left(\mu_{ik}\right)}^{\alpha }\text{,} \end{array}$$

where 1(*x*_*lj*_=*x*_*ij*_)=1 if *x*_*lj*_=*x*_*ij*_, where 1(*x*_*lj*_ ≠ *x*_*ij*_)=0 if *x*_*lj*_ ≠ *x*_*ij*_.*N*_*x*_*ij*__ is computed in the equation (14) as follows:

(14) $$\begin{array}{c} N_{x_{ij}}=\overset{n}{\underset{i=1}{\sum }}{\left(\mu_{ik}\right)}^{\alpha }\text{.} \end{array}$$

#### 2.2.4. Attribute Weight of Categorical Data

Let *W*=[*w*_1_^*r*^, *w*_2_^*r*^, ⋯,*w*_*p*_^*r*^, *w*_(*p*+1)_^*c*^, *w*_(*p*+2)_^*c*^, ⋯,*w*_*m*_^*c*^]^*T*^ be the weights for *m* attributes. Superscript *c* denotes weight for categorical attributes *W*^*C*^=[*w*_(*p*+1)_^*c*^, *w*_(*p*+2)_^*c*^, ⋯,*w*_*m*_^*c*^]^*T*^.Assuming *N*_*a*_*kj*_^*t*_1_^_(*t*_1_=1, 2, ⋯, *n*_*l*_) and *N*_*a*_*kj*_^*t*_2_^_(*t*_1_=1, 2, ⋯, *n*_*l*_) are data point numbers in Dataset *X*_*i*_(*i*=1, 2, ⋯, *n*) with the value *a*_*j*_^*t*_1_^, *a*_*j*_^*t*_2_^ for the *j*^*th*^(*j*=(*p*+1), (*p*+2), ⋯, *m*) attribute that belongs to cluster *k*(*k*=1, 2, ⋯, *C*), respectively. *N*_*a*_*j*_^*t*_1_^_ and *N*_*a*_*j*_^*t*_2_^_ are data point number in Dataset X_i_ with *a*_*j*_^*t*_1_^and *a*_*j*_^*t*_2_^ for the *j*^*th*^ attribute in all clusters, respectively. Based on providing the number of formula such as (2) and (3), the weight of categorical attribute *A*_*j*_(*j*=(*p*+1), (*p*+2), ⋯, *m*) can be calculated by weighting distance*ϑ*(*a*_*j*_^*t*_1_^, *a*_*j*_^*t*_2_^). Thus, the weight of attribute *A*_*j*_(*j*=(*p*+1), (*p*+2), ⋯, *m*) in *m* categorical attributes is as shown in the equation (15) as follows-

(15) $$\begin{array}{c} w_{j}^{c}=\frac{\sum_{t_{1},t_{2}=1}^{n_{l}}\vartheta \left(a_{j}^{t_{1}},a_{j}^{t_{2}}\right)}{n_{l}}\text{.} \end{array}$$

The weighted distance between *a*_*j*_^*t*_1_^ *and* *a*_*j*_^*t*_2_^ is given in equation (16) as follows:

(16) $$\begin{array}{c} \vartheta \left(a_{j}^{t_{1}},a_{j}^{t_{2}}\right)=\overset{C}{\underset{k=1}{\sum }}\left|\frac{N_{a_{kj}^{t_{1}}}}{N_{a_{j}^{t_{1}}}}-\frac{N_{a_{kj}^{t_{2}}}}{N_{a_{j}^{t_{2}}}}\right|\text{.} \end{array}$$

#### 2.2.5. Fuzzy Centre for Categorical Data Objective Function

We will apply the common objective function in the FCM algorithm [5], as presented in equation (17) as follows:

(17) $$\begin{array}{c} J=\overset{C}{\underset{k=1}{\sum }}\overset{n}{\underset{i=1}{\sum }}{\left(\mu_{ik}\right)}^{\alpha }d\left(X_{i},V_{k}\right)\text{.} \end{array}$$

When a dataset only has numeric attributes, the similarity is measured by the square of Euclidean distance. When a data set has mixed attributes of numerical and categorical data types, the similarity measure needs to incorporate weights of attributes to various cluster centers. Assuming a dataset *X*={*X*_1_, *X*_2_, ⋯, *X*_*n*_} has both numerical and categorical attributes. They belong to *C* clusters. Partition matrix *U*_*n*×*c*_ indicates the fuzzy membership degree of data *i* to the *k*th cluster. *μ*_*ik*_ is an element in the partition matrix *U*_*n*×*c*_ and subject to condition given in equation (18) as follows-

(18) $$\begin{array}{c} \overset{C}{\underset{k=1}{\sum }}\mu_{ik}=1,0\leq \mu_{ik}\leq 1\text{.} \end{array}$$

Their corresponding cluster center set is as given in equation (19) as follows-

(19) $$\begin{array}{c} V=\left[V_{1},\cdots {,V}_{k},\cdots ,V_{c}\right]\text{.} \end{array}$$

Each cluster center *V*_*k*_(*k*=1, 2, ⋯, *C*), includes numerical and categorical attributes and can be represented as in equation (20)

(20) $$\begin{array}{c} V_{k}=\left[v_{i1}^{r},v_{i2}^{r},\cdots ,v_{ip}^{r},v_{i\left(p+1\right)}^{c},v_{i\left(p+2\right)}^{c},\cdots ,v_{im}^{c}\right]\text{.} \end{array}$$

The weights for m attributes is given in equation (21):

(21) $$\begin{array}{c} W={\left[w_{1}^{r},w_{2}^{r},\cdots ,w_{p}^{r},w_{\left(p+1\right)}^{c},w_{\left(p+2\right)}^{c},\cdots ,w_{m}^{c}\right]}^{T}\text{,} \end{array}$$

where elements *p* with superscript *r* and *p* with superscript *c* are numeric values and categorical values respectively. The common objective function is given in equation (22)

(22) $$\begin{array}{c} J\left(U,V,W\right)=\overset{C}{\underset{k=1}{\sum }}\overset{n}{\underset{i=1}{\sum }}\mu_{ik}^{\alpha }d_{w}^{2}\left(X_{i},V_{k}\right)=\overset{C}{\underset{k=1}{\sum }}\overset{n}{\underset{i=1}{\sum }}\mu_{ik}^{\alpha }{\left\|X_{i}-V_{k}\right\|}_{w}^{2}. \end{array}$$

The common objective function is represented in equation (23) as follows:

(23) $$\begin{array}{c} J\left(U,V,W\right)=J^{r}\left(U,V,W\right)+J^{c}\left(U,V,W\right)\text{.} \end{array}$$

**Proof**

J  (*U*, *V*, *W*)=∑_*k*=1_^*C*^{*μ*_*ik*_^*α*^[∑_*i*=1_^*n*^[*W*‖*X*_*i*_ − *V*_*k*_‖]^2^]}=∑_*k*=1_^*C*^{*μ*_*ik*_^*α*^[∑_*i*=1_^*n*^∑_*j*=0_^*m*^[*w*_*j*_‖*x*_*ij*_ − *v*_*kj*_‖]^2^]}=∑_*k*=1_^*C*^{*μ*_*ik*_^*α*^[∑_*i*=1_^*n*^(∑_*j*=0_^*p*^(*w*_*j*_‖*x*_*ij*_ − *v*_*kj*_‖)^2^+∑_*j*=*p*+1_^*m*^(*w*_*j*_‖*x*_*ij*_ − *v*_*kj*_‖)^2^)]}=∑_*k*=1_^*C*^{*μ*_*ik*_^*α*^[∑_*i*=1_^*n*^∑_*j*=0_^*p*^(*w*_*j*_‖*x*_*ij*_ − *v*_*kj*_‖)^2^+∑_*i*=0_^*n*^∑_*j*=*p*+1_^*m*^(*w*_*j*_‖*x*_*ij*_ − *v*_*kj*_‖)^2^]}=∑_*k*=1_^*C*^{*μ*_*ik*_^*α*^[∑_*i*=1_^*n*^(*w*^*r*^‖*X*_*i*_^*r*^ − *V*_*k*_^*r*^‖)^2^+∑_*i*=1_^*n*^(*w*^*c*^‖*X*_*i*_^*c*^ − *V*_*k*_^*c*^‖)^2^]}=∑_*k*=1_^*C*^∑_*i*=1_^*n*^*μ*_*ik*_^*α*^(*w*^*r*^‖*X*_*i*_^*r*^ − *V*_*k*_^*r*^‖)^2^+∑_*k*=1_^*C*^∑_*i*=1_^*n*^*μ*_*ik*_^*α*^(*w*^*c*^‖*X*_*i*_^*c*^ − *V*_*k*_^*c*^‖)^2^=*J*^*r*^(*U*, *V*, *W*)+*J*^*c*^(*U*, *V*, *W*)

According to the above computation, the distance *d*_*w*_^2^(*X*_*i*_, *V*_*k*_) is as given in equation (24) as follows-:

(24) $$\begin{array}{c} d_{w}^{2}\left(X_{i},V_{k}\right)=d_{w}^{2}\left(X_{i}^{r},V_{k}^{r}\right)+d_{w}^{2}\left(X_{i}^{c},V_{k}^{c}\right)\text{,}\\ d_{w}^{2}\left(X_{i}^{r},V_{k}^{r}\right)={\left\|X_{i}^{r}-V_{k}^{r}\right\|}_{w}^{2}={\left(w^{r}\left\|X_{i}^{r}-V_{k}^{r}\right\|\right)}^{2}=\overset{p}{\underset{j=1}{\sum }}{\left[w_{j}\left(x_{ij}-v_{kj}\right)\right]}^{2},\\ d_{w}^{2}\left(X_{i}^{c},V_{k}^{c}\right)=\frac{1}{N_{k}}\overset{n_{l}}{\underset{t=1}{\sum }}N_{a_{kj}^{t}}\delta \left(x_{ij}^{c},a_{j}^{t}\right)=\frac{1}{N_{k}}\overset{n_{l}}{\underset{t=1}{\sum }}\left(N_{a_{kj}^{t}}\times \frac{1}{C}\left(\overset{C}{\underset{p=1}{\sum }}\left|\frac{N_{x_{ij},k}}{N_{x_{ij}}}-\frac{N_{a_{kj}^{t}}}{N_{a_{j}^{t}}}\right|\right)\right). \end{array}$$

#### 2.2.6. The Procedure of Applying the MD-MWFCM Algorithm

Let the dataset of biomedicine be *X*={*X*_1_, *X*_2_, ⋯, *X*_*n*_}. For a data point X_i_(i=1, 2, ⋯, n) having m features *m*={*A*_1_, *A*_2_, ⋯, *A*_*m*_}, the feature data set can be represented as *X*_*i*_={*x*_*i*1_, *x*_*i*2_, ⋯, *x*_*im*_}. The mixed numeric and categorical feature data set is represented as: *X*_*i*_=[*x*_*i*1_^*r*^, *x*_*i*2_^*r*^, ⋯, *x*_*ip*_^*r*^, *x*_*i*(*p*+1)_^*c*^, *x*_*i*(*p*+2)_^*c*^, ⋯, *x*_*im*_^*c*^](*i*=1, 2, ⋯, *n*); weight *W*=[*w*_1_, *w*_2_, ⋯,*w*_*m*_]^*T*^ represents the weight of a feature for the a biomedical clusters C={C_1_, C_2_, ⋯, C_c_}. This weight needs to be merged into the corresponding feature data set *W*=[*w*_1_^*r*^, *w*_2_^*r*^, ⋯,*w*_*p*_^*r*^, *w*_(*p*+1)_^*c*^, *w*_(*p*+2)_^*c*^, ⋯,w_m_^c^]^T^. The corresponding feature fuzzy membership is represented as a matrix U ∈ R^C×n^($\tilde{U}\in {\left[\mu_{ik}\left(X_{i}\right)\right]}_{i=1,2,\cdots ,n;k=1,2,\cdots ,C}$) under the following constraints given in equation (25).

(25) $$\begin{array}{c} \overset{C}{\underset{k=1}{\sum }}\mu_{ik}\left(X_{i}\right)=1,0\leq \mu_{ik}\left(X_{i}\right)\leq 1, \end{array}$$

where *μ*_ik_(X_i_) represents the fuzzy membership of biomedical data point X_i_(i=1, 2, ⋯, n) to the cluster *k*(*k*=1, 2, ⋯, *C*). In addition to using the original formula in the FCM algorithm to compute the center of symptom j in biomedical cluster k for numeric symptom data of dataset *X*_*i*_^*r*^=[*x*_*i*1_^*r*^, ⋯, *x*_*ij*_^*r*^, ⋯,*x*_*ip*_^*r*^](i=1, 2, ⋯, n; j=1, 2, ⋯, p), the MD-MWFCM algorithm will also calculate the fuzzy membership *μ*_ik_ for *r* both numerical and categorical feature data. Each cluster center V_k_ can be expressed as in equation (24) and the fuzzy membership is as given in equation (26) as follows-

(26) $$\begin{array}{c} v_{kj}^{r}=\frac{\sum_{i=1}^{n}\mu_{ik}^{\alpha }x_{ij}^{r}}{\sum_{i=1}^{n}\mu_{ik}^{\alpha }}\left(j=1,2,\cdots ,p\right)\\ \mu_{ik}=\frac{1}{\sum_{t=1}^{C}{\left(d\left(X_{i},V_{k}\right)/d\left(X_{i},V_{t}\right)\right)}^{1/\alpha -1}}, \end{array}$$

where d(X_i_, V_k_) and d(X_i_, V_t_) is the dissimilarity measure between each biomedical data point X_i_(i=1, 2, ⋯, n) and each cluster center V_k_(k=1, 2, ⋯, C; k ≠ t) and V_t_(k=1, 2, ⋯, C; t ≠ k). The parameter *α* is a fuzzy coefficient exponent for fuzzy degree of partition matrix U ∈ R^C×n^. To overcome the limitation of the FCM method in over sensitivity to initial cluster centers location, MD-MWFCM uses the minimum threshold method to initiate the cluster centers. First, it randomly locates two biomedical data points X_x_, X_y_(x, y=1, 2, ⋯, n; x ≠ y) into a C_1_. Then, it partitions the rest of the X_i_(i=1, 2, ⋯, n; i ≠ x, i ≠ y) according to the result of the dissimilarity measure d_w_(X_i_, X_x_) or d_w_(X_i_, X_y_), where the function d_w_(X_i_, X_x_) and d_w_(X_i_, X_y_) denotes comparison of similarity between X_i_ and X_x_ or X_y_.Assuming *D* as the threshold value for the dissimilarity measure, if d_w_(X_i_, X_x_) < *D* or d_w_(X_i_, X_y_) < *D*, then we allocate X_i_ into the cluster C_1_, otherwise allocate X_i_ into a new data cluster. We repeat this partition process until all biomedical data belong to certain clusters. A seven steps flowchart in implementing the MD-MWFCM algorithm is shown in Figure 1

The steps of the algorithms are as follows

Step 1. Input a normalized biomedical data X_i_={x_i1_, x_i2_, ⋯, x_im_}(i=1, 2, ⋯, n). Select the maximum iteration number max_Iteration, a cluster number C, a sensitivity threshold value *ε*, a threshold value *D* of minimum threshold method, and fuzzy coefficient *α*. Initialize fuzzy membership of the feature data points $\tilde{U}\in {\left[\mu_{ik}\left(X_{i}\right)\right]}_{i=1,2,\cdots ,n;k=1,2,\cdots ,C}$.
Step 2. Select the initial cluster center using minimum threshold method.
  Step 2.1. Randomly allocate two biomedical data points X_x_, X_y_(x, y=1, 2, ⋯, n; x ≠ y) into a cluster C_1_.
  Step 2.2. Compute the dissimilarity of the rest of the biomedical data point X_i_(i=1, 2, ⋯, n; i ≠ x, i ≠ y) with the original two data points X_x_ and X_y_ using the formulae (21)–(23). d_w_(X_i_, X_x_)=d_w_^2^(X_i_^r^, X_x_^r^)+d_w_^2^(X_i_^c^, X_x_^c^)d_w_(X_i_, X_y_)=d_w_^2^(X_i_^r^, X_y_^r^)+d_w_^2^(X_i_^c^, X_y_^c^) If d_w_(X_i_, X_x_) < *D* or d_w_(X_i_, X_y_) < *D*, allocate X_i_ into biomedical cluster C_1_, otherwise allocate X_i_ into a new cluster.
  Step 2.3. Repeat Step 2.2 until every data X_i_(i=1, 2, ⋯, n) has been allocated into C clusters.
  Step 2.4. If k=C, go to Step 2.5. If k ≠ C, change threshold value D and return to Step 2.1.
  Step 2.5. Calculate the initial cluster center V_k_=[v_i1_^r^, ⋯, v_ip_^r^, v_i(p+1)_^c^, ⋯, v_im_^c^](k=1, 2, ⋯, C) for each cluster using equations (24) and (11).
Step 3. Use the cluster centers V_k_(k=1, 2, ⋯, C) calculated in Steps 2.5 as the initial cluster centers V_k_^(0)^(k=1, 2, ⋯, C). Define the iteration count number l=1.
Step 4. Compute fuzzy membership of the feature data points U ∈ R^C×n^ by the equation (27), adding the iteration count number l.
  (27) $$\begin{array}{c} \mu_{ik}^{\left(l\right)}={\left[\overset{C}{\underset{t=1}{\sum }}{\left(\frac{d_{w}^{2}\left(X_{i},V_{k}^{\left(l-1\right)}\right)}{d_{w}^{2}\left(X_{i},V_{t}^{\left(l-1\right)}\right)}\right)}^{\frac{1}{\;\alpha -1}}\right]}^{-1}. \end{array}$$
Step 5. Compute cluster centers V_k_^(l)^=[v_i1_^r^, ⋯,v_ip_^r^, v_i(p+1)_^c^, ⋯,v_im_^c^]^(l)^(k=1, 2, ⋯, C) with equations (24) and (11) for numeric and categorical feature data.
Step 6. Compute feature weights W^(l)^=[w_1_, w_2_, ⋯,w_m_]^(l)T^for numeric feature data using equation (28) and categorical feature data using equation (29).
  (28) $$\begin{array}{c} w_{j}^{r}={\left[\overset{m}{\underset{t=1}{\sum }}\frac{\sum_{k=1}^{C}\sum_{i=1}^{n}\mu_{ik}^{\alpha }{\left(X_{ij}-V_{kj}\right)}^{2}}{\sum_{k=1}^{C}\sum_{i=1}^{n}\mu_{ik}^{\alpha }{\left(X_{it}-V_{kt}\right)}^{2}}\right]}^{-1},\left(t=1,2,\cdots ,p;j=1,2,\cdots ,p\right)\\ w_{j}^{c}=\frac{\sum_{t_{1},t_{2}=1}^{n_{l}}\vartheta \left(a_{j}^{t_{1}},a_{j}^{t_{2}}\right)}{n_{l}}\left(t=1,2,\cdots ,p;j=1,2,\cdots ,p\right). \end{array}$$
Step 7. Judge objective function value J(U, V, W) using formula (20). If |J^(l)^(U, V, W) − J^(l − 1)^(U, V, W)| > *ε* or l <  max   _*Iteration*, return to Step 4 and increase l=l+1. Otherwise, conclude.

## 3. Research Method

### 3.1. Data Description

Three datasets were used in the experiment and were all exported from the UCI Machine Learning Repository (https://archive.ics.uci.edu/ml/datasets.php). These include an Iris data set with pure numerical data, a Soybean data set with pure categorical data and a heart disease data set with mixed numeric and categorical data. The Iris data set has only four numeric attributes (sepal length, sepal width, petal length and petal width) and contains 150 data points equally in three clusters: iris Setosa (50), iris Versicolour (50), and iris Virginica (50). Since all attributes of the data set are numeric, only numeric objective function J^r^(U, V, W) is applied in the MD-MWFCM. The Soybean data set has all 35 categorical attributes (date, plant-stand, precip, temp, hail, crop-hist, area-damaged, severity, seed-tmt, germination, Plant-growth, leaves, leafspots-halo, leafspots-marg, leafspot-size, leaf-shread, leaf-malf, leaf-mild, stem, lodging, stem-cankers, canker-lesion, fruiting-bodies, external decay, mycelium, int-discolor, sclerotia, fruit-pods, fruit spots, seed, mold-growth, seed-discolor, seed-size, shriveling, roots) and 47 data points. The data points are grouped into four clusters: Diapor the Stem Canker (10), Charcoal Rot (10), Rhizoctonia Root Rot (10) and Phytophthora Rot (17). Only categorical objective function J^c^(U, V, W) is needed to cluster all categorical data attributes.

### 3.2. Experiment Setup

To implement the MD-MWFCM clustering algorithm, data initialization in Step 1 included the folloiwng: setting the maximum iteration number max   _Iteration = 10000, the cluster number C to be 3, 4 and 2 for Iris, Soybean, and Heart Disease data sets, respectively (see Table 1), the sensitivity threshold value *ε* = 0.0001, the threshold value D = 2 and fuzzy coefficient *α* ∈ [1.0,10.0] (see Table 1). Initialize fuzzy membership values *μ*_ik_(X_i_) ∈ (0.0, 1.0)(i = 1, 2, ⋯, n; k = 1, 2, ⋯, C) for random function under the constraint ∑_k=1_^C^*μ*_ik_(X_i_) = 1. The MD-MWFCM clustering algorithm was run for each data set. Since the three datasets are standard datasets which have been normalized in the UCI Machine Learning Repository, in Step 1 (see Figure 1), the data points with the relevant attributes are input parameters to run the MD-MWFCM clustering algorithm for each data set (Iris, Soybean and Heart Disease, respectively) (See Table 1). Steps 2 to 7 (Figure 1) are executed automatically by the software programs. Each dataset was run 100 times for each value of the fuzzy coefficient {1.0, 1.1, 1.2,… 10.0} to select the optimal true positive value as the output result at each value of the fuzzy coefficient (see Table 1). Each output result represents a cluster centre. All experiments are implemented on a Microsoft ThinkPad E450 PC with 8G byte main memory and Microsoft Windows XP operating system. The algorithms were implemented in Visual C++ programming language. Input parameters of each dataset for executing the MD-MWFCM clustering algorithm are given in Table 2

### 3.3. Performance Measurement

The performance of the algorithms is accessed by clustering accuracy (r) as given in equation (29)

(29) $$\begin{array}{c} r=\frac{\sum_{k=1}^{c}a_{k\;}}{n}, \end{array}$$

where a_k_ is the data point number in the kth(k=1, 2, ⋯, C) cluster with true positive value. n is the total number of the data set. A higher value of r suggests better performance of the algorithm.

### 3.4. Result and Discussion

#### 3.4.1. The Performance of the MD-MWFCM for Mixed Data

The MD-MWFCM algorithm have achieved the highest clustering accuracy for three data sets compared with the four common clustering algorithms: k-prototypes, SBAC, KL-FCM-GM and IWKM. The value of r is 0.967 in clustering the numeric Iris data set by the MD-MWFCM. This is 14.8%, 59.4%, 63.2% and 14.5% higher than k-prototypes, SABC, KL-FCM-GM and IWKM algorithms (see Table 3). For the categorical Soybean dataset, *r* of the MD-MWFCM is 1, achieving clear grouping of clusters. It outperformed k-prototypes, SABC, KL-FCM-GM and IWKM algorithms by 14.4%, 38.3%, 9.7% and 9.2%, respectively (see Table 4). Clustering accuracy *r* was 0.779 for the heart disease dataset using the MD-MWFCM (see Table 5). This was 23.3%, 23.4%, 12.6%, and 12.6% more clustering accuracy than that of the k-prototypes, SABC, KL-FCM-GM, and IWKM algorithms. The comparison of the maximum accuracy achieved by five clustering algorithms for the Iris data set is as shown in Table 1:

The comparison of the maximum accuracy achieved by five clustering algorithms for the Soybean data set is shown in Table 3.

The comparison of the maximum accuracy achieved by five clustering algorithms for the Heart Disease data set is given in Table 4

A comparison of the common algorithm for clustering mixed categorical and numeric data set is shown in Table 5

The k-prototypes algorithm has its advantage in a global optimal search, but falls short in losing information about multiple memberships of a data point (refer Table 5). The SBAC algorithm uses the same agglomerative algorithm to construct a dendrogram to display the similarity (or difference) level of a pair of data points with numeric or nominal attributes. Its limitation is to give larger weight to uncommon attributes which may lead to its unreasonable significance in clustering. The KL-FCM-GM algorithm with Gath-Geva theory is more suitable for clustering numeric data with Gath distribution. Although the IWKM algorithm performs relatively better than k-prototypes, SBAC and KL-FCM-GM algorithms in mixed numeric and categorical data types, it is over sensitive to cluster center initialization for different attributes. The proposed MD-MWFCM clustering algorithm has shown its higher performance than these clustering algorithms for mixed data. It has introduced a different representation of cluster centers for different data types, i.e., numeric data center for numeric data type and categorical data center for the categorical data type. For numeric and categorical data in biomedicine, techniques for dealing with categorical data are usually more difficult than those for numeric data. The k-modes, as a classical categorical clustering method has demonstrated its advantages. Compared with k-modes, the MD-MWFCM clustering algorithm has been improved in following aspects. First is that fuzzy membership has be applied in MD-MWFCM clustering algorithm to reflect the relation degree of a data point to each cluster center while k-modes only considers hard fuzzy partition. Moreover, fuzzy membership also has been both combined into the dissimilarity measurement and objective function process with weighting. The MD-MWFCM clustering algorithm uses different dissimilarity measure individually for numeric and categorical data in a cluster. This can fully use fuzzy membership in clustering vague data across the boundaries of clusters. The objective function calculates dissimilarity by data types and weights of attributes in the iteration of clustering. In the partitioned clustering algorithm, the initial position of the cluster center has a significant impact on the clustering results. The randomness of this initialization method is too strong, which leads to great fluctuation of clustering effect, and the same clustering results are difficult to reproduce. The improved cluster center initialization method in MD-MWFCM clustering algorithm is proposed. The initial centers from the results in the minimum threshold method can help avoiding the randomness problem of initial cluster centers in a random way. The minimum threshold method can fix the cluster centers in a possible defined range. All these have enabled the MD-MWFCM to outperform the other four algorithms in clustering all three datasets, only numerical, only categorical, and mixed numerical and categorical datasets.

*(1) The Optimal Fuzzy Coefficient α Value in Accordance with the Maximum Clustering Accuracy* **r**. When *α* ∈ [1.0, 3.0], the Iris dataset achieved its optimal clustering accuracy of 0.967 as shown in Figure 2).

When *α* ∈ [1.0,10.0], the Soybean dataset achieved its optimal clustering accuracy of 1.000 as shown in Figure 3

When *α* ∈ [1.0,10.0], the heart disease dataset achieved its optimal clustering accuracy of 0.779 as shown in Figure 4

Because overlap degree between the clusters in a data set is mainly impacted by the fuzzy coefficient *α*, the degree of overlap reflects the distribution of data points in each cluster which can be indicated by calculating clustering accuracy *r*. Therefore, the clustering accuracy *r* in the MD-MWFCM algorithm is mainly impacted by *α* (see Figures 2–4) instead of the numerical value fluctuation in the Iris dataset or the categorical values in the Soybean dataset. It has been an ongoing challenge to select the value of *α* in fuzzy data analysis. Several researchers have attempted to address this challenge. These attempts all use mathematical programming in selecting the values of a fuzzy correlation coefficient, and it is not easy to propose further applications for researchers who don't have a strong mathematical background. The authors suggested that the optimal clustering accuracy *r* is achieved when *α* is within 10.0, especially when *α* ∈ [1.5, 2.5] [14]. Our study has contributed empirical evidence to support their suggestion. By starting the experiment with the *α*value of 1.0, and incrementing it at 0.1 interval, we can accurately pinpoint the value *α* with accuracy to 0.1 for the corresponding optimal clustering accuracy *r*. Every dataset has its own optimal fuzzy coefficient value suggested by the corresponding optimal clustering accuracy *r* (see Figures 2–4). Before achieving the aim of the objective function, the clustering accuracy *r* is not substantially impacted by the changing value of fuzzy coefficient *α*; this suggests that the performance of the MD-MWFCM algorithm is reasonably stable. According to article [3], one performance criteria of a clustering algorithm is its convergence speed of the clustering algorithm. According to article [4], being able to achieve the optimal clustering accuracy with *α* < 10.0, is an indication that the objective function can converge at reasonable speed. The convergence was achieved when *α*=1.5 for the Iris dataset (Figure 2), *α* ∈ [1.1, 1.2] for the Soybean dataset (Figure 3) and *α*=2.2 for the Heart Disease dataset (Figure 4). Because the objective function achieved convergence with small fuzzy coefficient values (*α* < 3.0) in all three data sets, it suggests that the MD-MWFCM algorithm has high performance speed.

## 4. Conclusion

To address the limitations of FCM, this study proposes a novel multiple weighted fuzzy C-means for mixed data (MD-MWFCM) clustering algorithm. The MD-MWFCM algorithm presents a novel clustering FCM algorithm by treating numeric and categorical data individually with their respective cluster center representation, dissimilarity measurement and objective function aspects. For cluster center representation, mean is used for numeric data and fuzzy center is used for categorical data. Based on the different cluster center representations, it uses different dissimilarity measurement methods to compute the distance of a data point to various cluster centers. For dissimilarity, numeric data are calculated by the distance and weight of a data point to each cluster centre, categorical data are measured by the frequency of occurrence and weight of a data point to a cluster. The objective function is computed by the dissimilarity measurement. Moreover, the MD-MWFCM algorithm is improved from cluster center initialization through the minimum threshold method. The proposed algorithm is implemented on three standard datasets (Iris dataset, soybean dataset and heart disease) and compared with other clustering algorithms. Results showed that the efficiency of the MD-MWFCM approach in improving the performance of a pure numerical dataset (Iris dataset) are individually up to 14.8%, 59.4%, 63.2% and 14.5% compared with k-prototypes, the similarity-based agglomerative clustering (SBAC) algorithm, Kullback–Leibler Fuzzy C-means algorithm for Gauss-Multinomial-distributed data (KL-FCM-GM), and the improved weighting k-Mean clustering algorithm (IWKM). Results with pure categorical dataset (Soybean dataset) are individually up to 14.4%, 38.3%, 9.7%, and 9.2%. In the same way, the improvement of the MD-WFCM algorithm in a mixed dataset (heart disease) is 23.3%, 23.4%, 12.6%, and 12.6%. The performance of the MD-WFCM algorithm has illustrated its useful application not only in a pure attribute dataset (numerical data or categorical data), but also, more importantly, in a mixed biomedical dataset.

## 5. Future Scope

In future, the ensemble clustering technique that deals with high-dimensional data and fuses multiple clustering results into a better clustering performance will be considered for the further improvement in clustering techniques.

## Figures and Tables

**Figure 1:** MD-MWFCM algorithm.

**Figure 2:** The optimal accuracy (**r**) of the MD-MWFCM with varying fuzzy coefficient *α* for the Iris dataset.

**Figure 3:** The optimal accuracy (**r**) of the MD-MWFCM with varying fuzzy coefficient *α* for the Soybean dataset.

**Figure 4:** The optimal accuracy (**r**) of the MD-MWFCM with varying fuzzy coefficient *α* for the heart disease dataset.

**Table 1:** Comparison of the maximum accuracy achieved by five clustering algorithms for the Iris data set.

Algorithm	Clustering accuracy (r)
k-prototypes	0.819
SBAC	0.373
KL-FCM-GM	0.335(*α*=1.1)
IWKM	0.822
MD-MWFCM	0.967 (*α*=1.5)

**Table 2:** Input parameters of each dataset for executing the MD-MWFCM clustering algorithm.

Input parameter	Iris dataset	Soybean dataset	Heart disease dataset
*n* (Sample size)	150	47	303
*m* (Attribute number)	4	35	13
*C* (Cluster number)	3	4	2
*α* (Fuzzy coefficient)	[1.0, 10.0]	[1.0, 10.0]	[1.0, 10.0]
*m* − *p* (Categorical attribute number)	0	35	8
*Dom*(*A*) (Categorical attribute domain)	See iris dataset	See soybean dataset	See heart disease dataset
The value of each data point	See UCI machine learning repository		

**Table 3:** Comparison of the maximum accuracy achieved by five clustering algorithms for the Soybean data set.

Algorithm	Clustering accuracy (*r*)
k-prototypes	0.856
SBAC	0.617
KL-FCM-GM	0.903(*α*=1.8)
IWKM	0.908
MD-MWFCM	1.000(*α* ∈ [1.1,1.2])

**Table 4:** Comparison of the maximum accuracy achieved by five clustering algorithms for the heart disease data set.

Algorithm	Clustering accuracy (*r*)
k-prototypes	0.546
SBAC	0.545
KL-FCM-GM	0.653(*α*=1.3)
IWKM	0.653
MD-MWFCM	0.779(*α*=2.2)

**Table 5:** A comparison of the common algorithm for clustering mixed categorical and numeric data set.

Clustering method	Analysis	Limitation
k-prototypes [10]	Step 1. Select several data points as the initial cluster centres randomly	Data can only be allocated into one cluster, losing information about multiple membership; Sensitive to initialization of cluster centres; No discretion of varying weights of an attribute in different clusters
	Step 2. Allocate the rest data points with the highest similarity to the relevant cluster centre	
	Step 3. Update the cluster centres after each data allocation	
	Step 4. Recalculate the dissimilarity of each data point to each cluster centre	
	Step 5. Repeat steps 2 to 4 until reaching the optimal cluster allocation	

SBAC [11]	Step 1. Create a cluster that contains a pair of data points with the highest similarity	Uses the same method to measure both numerical and categorical data; Sensitive to initialization of cluster centres; No discretion of varying weight of an attribute in different clusters
	Step 2. Add another data point and compare its similarity with the initial two data points. If the similarity is higher than that of the two original ones, add to the cluster; otherwise treat the data as a new cluster centre	
	Step 3. Repeat Step 2 until all data points have been located to a cluster	
KL-FCM-GM [13]	Step 1. Use gath-geva theory to allocate fuzzy membership of all data points	Sensitive to initialization of fuzzy membership
	Step 2. Update weight of each data point in the allocated clusters	
	Step 3. Retest the distance of data point to cluster centre	
	Step 4. Estimate the cluster distribution parameters of gath-geva formula again	
	Step 5. Repeat steps 1 to 4 until the objective function has reached the stop condition	

IWKM [14]	Step 1. Select several data points as the initial cluster centres randomly and assign weight to each	Sensitive to initialization of cluster centres
	Step 2. Compute fuzzy membership matrix based on the values of the initial cluster centres and their weights obtained in Step 1	
	Step 3. Update cluster centres with the values of fuzzy membership matrix and weights in Step 2	
	Step 4. Update the weights with the values of fuzzy membership matrix and cluster centres in Step 3	
	Step 5. Repeat steps 2 to 4 until the objective function has reached the stop condition	

## Data Availability

The data will be shared on request to the corresponding author.
